# Construction and Application of Psychological Quality Assessment Model for College Students Based on Extensive Data Analysis

**DOI:** 10.1155/2022/7982808

**Published:** 2022-05-20

**Authors:** Ping Zou, Yanjun Wu, Jingdan Zhang

**Affiliations:** ^1^Department of Student Affairs, Hebei Normal University of Science and Technology, Hebei, Qinhuangdao, 066000, China; ^2^School of Urban Construction, Hebei Normal University of Science and Technology, Hebei, Qinhuangdao, 066000, China; ^3^School of Agronomy and Biotechnology, Hebei Normal University of Science and Technology, Hebei, Qinhuangdao, 066000, China

## Abstract

This paper constructs a platform framework for extensive data analysis of college students' psychological quality with the help of the thinking mode of big data and related technologies and proposes the construction principles, data sources, data processing methods, data platform construction, and platform application of big data analysis platform for college students' psychological quality assessment. This paper combines the application methods of big data technology, collects the management data related to the psychological quality assessment of college students, saves them into the system database with certain storage logic, and realizes the function of psychological quality assessment through the design of selected psychological quality assessment data, data management and data resource management and other parts based on the data results of extensive data analysis. This study provides some insights into the psychological quality assessment of college students. The strength of association between the variables of psychological quality assessment of college students changes over time, but the overall psychological structure is more stable. This stable psychological structure characteristic is conducive to constructing the policy of constant psychological education in large universities.

## 1. Introduction

As a product of psychological research, psychological quality is a localized concept proposed and developed by psychologists in the context of active quality education of students. Psychological quality is based on physiological conditions and internalizes externally acquired stimuli into stable, essential, and implicit psychological qualities that have basic, derivative, developmental and self-organizing functions and are closely related to adaptive, developmental, and creative behaviors. The psychological quality is the endogenous factor of their mental health, which has a significant direct and regulatory role in individual mental health. The psychological quality education course management system for college students is a sub-system embedded in the psychological quality education system, with course management as its primary goal. The cultivation and formation of sound psychological quality are vital to enhancing the individual's ability to adjust and adapt psychologically, prevent and alleviate psychological problems, and maintain mental health and personality integrity. At the same time, psychological quality is also an essential part of students' quality, constraining the cultivation and development of students' quality [1]. The starting point and focus of psychological quality research are to improve the overall quality of students.

Contemporary college students have active thoughts and a thirst for knowledge and are a social group with a high cultural level among the youth. Not only do they need solid theoretical knowledge, but also a healthy body and a good heart. The university stage is critical for most college students to develop gradually into physical and mental maturity [2]. It is also essential for college students to build progressively from immaturity to maturity. With the change of social model, the fierce competition of employment, the conflict of new ideas, especially the role of some undesirable social phenomena, have a more significant impact on the psychology of college students who are in adolescence and immature physical and mental development; meanwhile, with the rapid growth of science and technology and the increase of the speed of knowledge update, the psychological pressure of college students also increases and numerous psychological problems appear [3]. If college students are still immature psychologically, their moods fluctuate, and their psychological tolerance is weak, they cannot bear the impact of social competition and changes.

The survey results show that among nearly 130,000 college students' mental health survey, about 1/5 of them have poor mental health. The information shows that almost 1/4 of the college students in the college group have psychological disorders. With the accelerated pace of life, psychological disorders among college students have reached nearly 35%. Many surveys have found that the incidence of psychological disorders among college students has gradually increased and has reached almost 40.0%, among which the performance of mental problems is outstanding. According to an epidemiological survey in Jiangxi, 2/5 of college students have compulsive tendencies, and 1/3 of college students have hostile emotions. A study on college students' mental health shows that college students' psychological disorders ratio is 1 : 50, and the percentage of psychological conflicts is about 1 : 4. It is found that the high incidence of psychological disorders is among all college students. University students are the core group of social development. Their mental health level is related to social development and an essential indicator of the health status of the whole society. Therefore, the psychological condition of college students has become the focus of attention of experts in many fields.

Good psychological quality is an integral part of the overall quality of students and an essential part of the comprehensive development of school education, which plays a vital role in the personality development, learning ability, ideological quality, and realization of life value of college students [4]. However, due to the popularization of higher education and new media communication, college students have “hollow disease” to varying degrees, which affects the state and quality of college students' mental health to a certain extent and directly affects the quality of college talent cultivation. The research group combines the new characteristics, new needs, and new problems of the psychological development of college students in the new era, researches five majors, tries to introduce film and television art into the process of college students' psychological health education, explores the feasibility and effectiveness of film and television art appreciation to improve the psychological quality of college students, to build a new model of psychological health education that is integrated with and out of the classroom, and improves the psychological quality of college students comprehensively.

## 2. Related Works

The research on the psychological quality of students began with secondary school students, and the research on the psychological quality of college students has been actively developed since the 21st century. With the popularization and development of mental health education in colleges and universities, the research on the psychological quality of college students involved in psychological quality education has become more prosperous. Big data analysis planning needs to be done jointly using domain business orientation and data drive, i.e., in the extensive data analysis methodology of determining the number of analysis objectives, data understanding and preparation, modeling to the final application, etc., the analysis logic is designed from the decomposition of key business objectives, the statute analysis process does not stray beyond the goals and requirements of the problem, and the completeness of the integrated business value, data and execution conditions are transformed into a solvable data analysis process. The exploration of the psychological quality of college students is an objective requirement for the implementation of quality education in colleges and universities and a practical need to promote the psychological health of college students [5]. Therefore, the systematic exploration of the current characteristics and development rules of the psychological quality of contemporary college students can help to improve further the relevance and effectiveness of the psychological quality education of college students, and then optimize the psychological quality of college students, and finally promote the healthy development of college students' body and mind.

From the perspective of college students' psychological quality assessment, Parry D A compiled the original version of the college students' psychological quality scale based on the concept and structural components of psychological quality proposed byDavidson B I in the early days, with a total of 130 questions, consisting of three parts: cognitive subscale, personality subscale, and adaptation subscale [6]. Börner K believed that psychological quality is composed of cognitive ability, personality trait, interpersonal management, vocational ability, psychological motivation, learning psychology, and self-awareness [7].considered that psychological quality is a stable psychological characteristic consisting of seven specific dimensions: cognitive ability, personality traits, interpersonal management, vocational ability, psychological motivation, learning psychology, and self-awareness, and compiled a total of 133 questions based on this scale; Charmaz K considered that psychological quality of college students should be composed of two parts, namely, cognitive ability quality based on intelligence and mental health quality based on personality, and scored each of them in the assessment. Based on the previous study [8]. Williamson B compiled his questionnaire on the psychological quality of college students based on the social and psychological development characteristics of current college students and formed a formal questionnaire with 32 items through question screening, containing five aspects of interaction adaptation, network coping, cognitive patterns, emotional control and stress coping [9]. In summary, although the questionnaire on assessing the psychological quality of college students is rich in style, there are still significant problems.

First of all, previous studies mainly used general factor or dimensional models in preparing the questionnaire, using the results of each dimension or element to explain the overall psychological quality, ignoring to some extent that psychological quality as a higher-order factor itself has its characteristics and values. As the conceptual definition of psychological quality shows, it is a comprehensive psychological quality of an individual. Even from the fit indices of the existing reported models, the fit results are not satisfactory enough. The researchers failed to make further modifications on this basis, which makes people doubt the rationality of the theoretical model on which the scale is based. Secondly, college students' existing psychological quality questionnaires are scored mainly by adding up the scores of each question item, which ignores the differences between dimensions and does not consider the overall psychological quality, contrary to the connotation structure of psychological quality itself. Finally, most of the existing questionnaires were developed in the early days of psychological quality research, and the test methods were simple. Most questionnaires had too many questions and were too long, not conducive to large-scale group testing.

In recent years, two-factor models have been increasingly used in psychometric applications. Some researchers have examined the similarities and differences between traditional structural models and two-factor models and found that two-factor models are generally more consistent with the definition of conceptual structure and have better fitting results than traditional structural models, i.e., the use of two-factor models can better explain the rationality of the theoretical structure underlying questionnaire development, and therefore the application of two-factor models to a psychological quality structure is scientific and operational. Therefore, applying the two-factor model to the psychological quality structure is scientific and operational. Based on the above reasons, Brackett M A and Bailey C S carried out a new round of revision of the psychological quality questionnaire for college students revised by Hoffmann J D based on the theory of the two-factor model. Finally, they formed the existing 27-item psychological quality questionnaire for college students (simplified version) [10]. The empirical study showed that the cognitive quality dimension.

The psychological quality, personality quality, and adaptability dimensions are highly correlated with psychological quality in general, and the components are moderately associated with each other [11]. This indicates that the members of psychological quality are independent of each other and have a specific attribution, i.e., they are unified in the comprehensive psychological quality of psychological quality. In the validated factor analysis of psychological quality structure, the researchers compared the relevant data results of the traditional three-factor model, one-factor model, and second-order model. The two-factor model had the best fitting results (Snedden T R, Scerpella J) [12]. Therefore, this study will use the Psychological Quality Questionnaire for College Students (simplified version) as the assessment tool to examine the psychological quality questionnaire for college students.

Although the questionnaire was revised to consider the rationality of demographic distribution as much as possible, there were still some problems [13]. The questionnaire sample was taken from 18 colleges and universities (each in the eastern, central, and western regions, and three key and public institutions in each area), with 3,182 actual valid questionnaires; among them, 1,166 (36.64%) were male students, 1,887 (59.30%) were female students, and 129 (4.05%) were gender deficient (Ferrari M and Hunt C) [14]. Follow-up studies showed that there were significant gender differences and disciplinary category differences in the psychological quality of college students, with male students having a significantly higher psychological rate than female students and natural science majors having significantly higher psychological quality than humanities and social science majors (Foster K, Roche M, Delgado C) [15]. However, the premise of the comparison of differences between groups is that the scale has measurement equivalence, which is the only way to ensure that the comparison between groups has authenticity and validity [16]. Meanwhile, other studies have shown that the ability characteristics of students in different subject specialization types are significantly different, and it is reasonable to use different evaluation methods to measure their accurate levels (Kwan I, Dickson K, Richardson M) [17]. In response to the sample sampling in the revision process of this scale, the gender ratio of male and female students differed significantly. It was primarily concentrated in humanities and social science majors, and it was unknown whether the questionnaire had measurement equivalence across gender and disciplinary types. Therefore, the Psychological Quality Questionnaire for College Students (simplified version) in different gender and professional groups needs further empirical testing [18].

## 3. Methods

### 3.1. Research Design

Extensive data analysis is one of the critical performance characteristics of big data technology, and extensive data analysis has positively affected social development and market economy enhancement. In the psychological quality assessment of college students, comprehensive data analysis has also played an obvious value, bringing more accurate judgment to the psychological quality assessment of college students, allowing college students to learn to actively apply big data in the process of psychological quality assessment and to explore potential information resources of psychological quality assessment through big data. Big data analysis in the psychological quality assessment of college students has also played an obvious value, bringing more accurate judgment to the psychological quality assessment of college students, allowing them to learn to actively apply big data in the process of psychological quality assessment and to explore potential information resources of psychological quality assessment through big data. Due to the many advantages of big data technology, coupled with the lack of practical experience in psychological quality assessment of college students, college students have fully recognized extensive data analysis, and are actively finding the most appropriate psychological quality assessment path through comprehensive data analysis, to achieve the established psychological quality assessment goals.

### 3.2. Participants

The study followed the principle of whole-group random sampling, and four institutions were selected in the eastern, central, and western regions, including six key institutions and six non-key institutions, involving different types of institutions as far as possible, consisting of a total of 120 students, including 12 male students and 108 female students; the control group consisted of 120 students majoring in animation, art design, and cultural industry management, including The control group, consisted of 120 students majoring in animation, art design, and cultural industry management, of which 14 were male, and 106 were female. The differences in the psychological quality of college students are shown in Figure 1.

### 3.3. Measures

A combination of quantitative and qualitative, factual, and deliberative methods is used to evaluate students' school performance. The comprehensive assessment is divided into basic quality assessment and developmental quality assessment. The essential quality refers to students' moral, intellectual, physical, and aesthetic attributes formed in teaching and second class in the college. The developmental quality refers to the creative and practical qualities that students develop in their education in college.

The psychological quality questionnaire (simplified version) was administered to college students. The questionnaire consists of 27 items, including three sub-dimensions of cognitive quality, personality quality, and adaptive ability. It is scored on a 5-point scale, with options 1 to 5 indicating a range from very poor to very good. The higher the total score of the questionnaire, the better the individual's psychological performance. Studies have shown that the scale meets the existing psychometric standards for construct validity and calibration validity and has high homogeneous reliability and retest reliability. In the sample of this study, the Cronbach's coefficients of the overall questionnaire and the sub-dimensions were 0.938, 0.862, 0.836, and 0.889.

### 3.4. Design

The primary purpose is to do an excellent job of feedback of the psychological quality assessment of college students, to give timely feedback of various relevant information of the students to the thinking counselor or class teacher who is responsible for managing the students, and at the same time, to analyze various information records and produce reports and graphs [19]. The system is designed to provide a comprehensive and intuitive understanding of the student's information for the student's teachers. System structure: The system uses the B/S method to realize some functions and applications of the psychological assessment analysis and early warning system. System implementation: A relational database system is used to build a database to store basic information such as department, counselor, classroom teacher, and student, as well as information about the assessment system and related assessments. The software of psychological assessment analysis and early warning system for college students was developed using Apache HTTP and python technology.

The system mainly includes two functional modules: student self-assessment and teacher management. Students' self-assessment: used primarily for complete students' self-assessment according to their actual situation through various self-assessment scales in the system, and at the same time, they can talk with teachers through the form of the message; teachers' management: mainly used to view students' letter, view students' assessment and statistical analysis results. Teachers can connect to the website with a browser, view students' messages and respond to them, and view the results of student assessments and statistical analysis to understand the overall situation of students.

The course management system of psychological quality education for college students is embedded in the design, taking course management as the primary goal. The course management system must align with the overall destination of psychological quality education for college students and pay attention to the communication and connection with the teaching cultivation goal [20]. In addition, the opening and management of the curriculum must be based on the inherent components of psychological quality, taking into full consideration the cognitive factors, personality factors, and adaptability factors. Curriculum management needs to realize the classification and targeted management of the curriculum from the characteristics of the development of psychological quality education and the main psychological problems. To ensure the smooth construction of the designed psychological quality assessment system for college students based on extensive data analysis, we test the various functions of the assessment system, build the corresponding psychological quality education platform, objectively and realistically simulate the whole process of online learning and online training management, to test the various application functions of the psychological quality education course management system and accumulate experience for the implementation of the project. According to the results of the demand analysis of the above system design, to ensure the rationality of the logical structure of the college students' psychological quality education course management system, improve the development efficiency of the software system, and at the same time reduce the maintenance cost of the course management system, specific system design is carried out from three parts: hardware, database, and software, respectively, and the overall design scheme of the system is derived.

Among the three modules of the system design, the hardware module provides hardware support for the software functions and data storage. It provides an interactive interface for the user to ensure the implementation and output of the system functions. This design is based on the traditional hardware system for data communication transmission, storage, and processing. We optimize and modify the modules, such as the processor, to improve the system performance from the hardware perspective.

The data communication method used in the course management system in this paper is the dual-port RAM communication method. This communication method utilizes a dual-port RAM chip. The two sets of communication lines are relatively independent in the actual communication process, and the muffler control signals between the two processors are realized through interrupt logic [21]. In addition to the above two communication lines also need to access the read-write timing control line in the communication network to regulate the data transmission data and real-time communication.

The architecture and functions of the core processor of the management system represent and determine the development level of the system to a certain extent. In the paper, a model TMS320C6722B floating-point chip is selected to replace the traditional core processor chip with an enhanced CPU C67x+, which significantly improves speed, coding, and computing power while being compatible with the CPU device. The replacement and optimization of the processing chip increase the memory storage space and enables an efficient 4-stage instruction pipeline and single-cycle instructions.

Since the internal data storage capacity of the college students' psychological quality education course management system directly affects the data processing efficiency, the memory device needs to be optimized. The memory module is divided into three types: program memory, data memory, and resource memory, among which program memory is used to store the management program of the course and the monitoring program of course teaching, the data memory is used to save a series of data resources generated during the operation of the system function and the work of the program, and resource memory is mainly used to store the help of the psychological quality education course and the resource data that the user needs to save within a specific time. The resource memory is mainly used to store the psychological education course resources and the resource data that users need to keep within a particular time. The three different types of memory work and operate synergistically. The large-capacity memory can effectively mitigate program operation and data access conflicts when the program is cached [22]. All the memory device interfaces in the memory module are parallel 8-bit FLASH chips capable of reaching about 64 KB of access space. The maximum addressing space can be increased to 8 MB after expanding the memory address through pins.

The data output control module is divided into several aspects, such as LCD and keyboard control. The central performance of the LCD module is to display the content 128 × 64 dot matrix, point size 0.50 mm ×0.50 mm, point spacing 0.05 mm, can show four lines of character content. The control of the display module CMl2864ZK in the course management system must fully comply with the timing requirements of the liquid crystal controller read and write, and its read and write parameters are shown in Table 1. And the keyboard in the course management system uses a four × four matrix keyboard, using four I/O lines as the row line, four I/O lines as the column line composed of the keyboard. The control of the course management program is achieved through the keyboard's power. To ensure the rationality of the logical structure of the college students' psychological quality education course management system, enhance the development efficiency of the software system, and at the same time reduce the maintenance cost of the course management system, the specific system design is carried out in three parts: hardware, database, and software, respectively.

### 3.5. Analysis

Descriptive statistics were performed on the data using SPSS 21.0 software to determine each question's mean, standard deviation, skewness, and kurtosis. Next, single-group validation factor analysis was performed, and standardized factor loadings were determined using Mplus 7.0 software; finally, morphological equivalence, weak equivalence, substantial equivalence, and strict equivalence tests were performed sequentially. It is generally accepted that the model achieves a good level of fit when RMSEA ≤0.08, CFI ≥0.90, TLI ≥0.90, and SRMR ≤0.08. It has been shown that the chi-square test results are easily affected by the sample size. When the sample size is sufficiently rich, significant difference results can be obtained even if the actual differences are slight. Therefore, this study used the difference in model fit indices CFI and TLI (i.e., ∆CFI and ∆TLI) to assess measurement equivalence. ∆CFI<0.01 and ∆TLI<0.01 indicate no significant difference between the two models, meaning equality can be accepted. We found that the overall psychological performance of the two groups of students was not significantly different and showed certain commonalities: compared to the non-artistic For the class students, the general psychological and adaptive qualities were higher and cognitive qualities were weaker for the art students; relative to the female students, the male students had more robust psychological and mental attributes and weaker adaptive abilities, while there was no significant difference between male and female students in terms of personality qualities. The two groups presented greater on the post-test by trying on the experimental group.

## 4. Results

### 4.1. Two Groups of Participants from Different Types of Institutions Were Studied, and Mathematical and Statistical Methods Analyzed the Data of the Test Indexes of the Experimental Group

We found that the overall psychological quality performance of the two groups of students was not significantly different and showed certain commonalities: compared to female students, male students had higher overall psychological quality and adaptability and poorer cognitive quality; compared to female students, male students had more robust psychological quality and mental quality and weaker adaptability, while there was no significant difference in personality quality between male and female students.

The overall psychological quality of students in both groups has been improved after receiving mental health education for college students, but the overall effect of the experimental group is significant; from the three dimensions, cognitive quality has been improved the most, followed by personality quality and adaptive ability; from the male and female gender, the improvement of female students is significantly better than male students [23]. It can be seen that by introducing college students to the teaching of mental health education courses, students' cognitive quality, personality quality, and adaptive ability were greatly improved, effectively improving the psychological quality of college students and highlighting the subtle effect of mental health education.

The “nurturing” function of the “cultural” part. The experiment did not significantly affect the cultivation of three aspects of college students' will qualities: toughness, decisiveness, and clarity of purpose. This is because cultivating college students will be a subtle and long-term strategy. The cultivation of will needs to be carried out throughout the students' academic life. The similarities and differences between the traditional structural model and the two-factor model were found, and it was found that the two-factor model was generally more consistent with the definition of conceptual structure, and the relevant results were better than the traditional structural model, i.e., the use of the two-factor model could better explain the rationality of the theoretical structure on which the questionnaire was developed, so the application of the two-factor model to the psychological quality structure was scientific and operational. Although the level of college students' psychological quality can be improved to a certain extent after a short period of training, if for specific psychological quality improvement, the more detailed targeted psychological quality assessment may need to be developed according to the target objects to adapt to the needs of different regions, different universities, and different individual students.

### 4.2. Big Data Analysis

Extensive data analysis is a series of analysis processes to maximize data value for specific domain application scenarios and obtain valuable decision-making information such as basic patterns, trends, and correlations. The cultivation and formation of sound psychological quality are essential for individuals to enhance their psychological adjustment and adaptability, prevent and alleviate psychological problems, and maintain their mental health and personality integrity. However, at the same time, big data analytics gradually reveals a situation of polarized knowledge, with data analysts lacking an in-depth understanding of domain business processes and domain personnel relatively lacking in knowledge of data analytics [24]. The traditional general extensive data analytics methodology only provides data mining application methods for practical application. Still, it lacks methodological guidance for integrating the essential domain business representation with the data processing process. Therefore, the planning of extensive data analysis needs to be done jointly by domain business orientation and data drive, i.e., in the process of determining the number of analysis objectives, data understanding, and preparation, modeling to final application in the extensive data analysis methodology, the analysis logic is designed from the decomposition of key business objectives, the analysis process does not stray beyond the goals and requirements of the problem, and integrates the business value, data and the completeness of the execution conditions, and transforms it into a solvable data model. The analysis process is transformed into an explicable data analysis process.

Based on the two-layer model of domain-oriented and platform-oriented extensive data analytics process, big data analytics can be realized by top-down goal decomposition, establishing domain-oriented extensive data analytics business process based on the analysis of interaction and combination relationship of business problems, and converting it into platform-oriented significant data analytics executable process instances according to model conversion rules and algorithms. Therefore, the extensive data analytic process processing framework is shown in Figure 2. The whole can be divided into user, processing, and execution layers, corresponding to the vast data analytical process's construction, mapping, and operation phases. The systematic exploration of the current characteristics of the psychological quality of contemporary college students and the law of development will help to improve further the relevance and effectiveness of college students' psychological quality education, thus optimizing the psychological quality of college students and ultimately promoting their healthy physical and mental development.

In the construction stage of the extensive data analysis process, this paper defines the tasks of complete extensive data analysis process as analysis module, significant data analysis process with analysis module as the smallest reusable unit, the analysis process editor of user layer provides reliable service column items, makes the analysis module presented to the user in the form of graphical elements, and defines a set of syntax, semantics and graphic relations of visual process description [25]. It is convenient for users to visually create and edit domain-oriented extensive data analysis business processes based on the analysis module and to realize the visualization of the parameters of each node in the process.

In the mapping stage of the extensive data analytic process, the conversion between process models is realized by the analysis module-based and model-driven model conversion algorithm. The domain-oriented big data analytical business process model is converted to the platform-oriented big data analytic process model, i.e., the model conversion algorithm is used, and according to the consistency correspondence between the user layer analysis module and the processing layer algorithm and the analysis model entity, the data analysis process from business description to data processing process.

In the operation phase of the extensive data analysis process, the platform-oriented big data analysis process model is instantiated into a process instance conforming to the execution platform specification according to the analysis module entity corresponding to each node and the input and output pattern information and parameter information. Good psychological quality is not only an essential part of the overall quality of individual students but also an essential element in the overall development of school education, which plays a vital role in the personality development, learning ability, ideological quality, and the realization of life values of college students. At this point, the user-defined domain-oriented big data analytic business process is transformed into a platform-oriented executable process, which can be executed in combination with the execution layer's computational resources, storage resources, and algorithm resources.

### 4.3. College Students' Psychological Quality

College students are free from their parents' care in their four-year critical schooling career, and they hope to become excellent and outstanding themselves through their efforts in this life stage, but this process inevitably has to face all kinds of worries such as study exams, friendship, love, employment pressure, exam pressure, work growth, etc. Students need to have a good psychological quality to face and solve all these pressures and worries. Since the internal data storage capacity of the psychological quality education course management system for college students directly affects the data processing efficiency, the memory device needs to be optimized. But at present, many college students do not have such good psychological quality and strong heart, the fact is that they have a variety of psychological problems, such as many students do not have self-confidence and have a potent inferiority complex, think they cannot do anything to do anything, do not dare to step out to brave practice, encounter difficulties and retreat; some students are shy and shy, do not dare to take the initiative and classmates and Some students are nervous and scared, afraid to take the initiative to interact with their classmates and teachers and ask for advice, they are in a closed state and do not have good interpersonal relationships; some students have the psychology of being out of touch and withdrawn and cannot integrate into the group life, some have the psychology of obsessive-compulsive anxiety and are always in fear. Living with such psychological problems and states is not conducive to the development of their lives, whether in school or society and is not conducive to a college student's full self-fulfillment and fulfilling and happy life.

At present, all major universities have their psychological assessment systems. They will accumulate specific data after the psychological assessment, increasing the accrued data year after year. After years of collection and convergence, the psychological assessment data become unique data resources. If not used for targeted analysis and utilization, it will only be dormant and worthless data and occupy hardware and software resources. Therefore, it is necessary to obtain the critical information hidden behind these data through specific technical means and analyze and utilize them at a higher level to play their proper value. The existing psychological assessment systems generally add, delete, modify, count, and query data. Still, they cannot discover the valuable knowledge and laws hidden in the data, nor can they predict whether college students will have various severe psychological problems based on the existing data. The application of data mining technology can make up for this problem to a certain extent. After years of use, the college counseling system has accumulated many students' psychological assessment data. If the relevant technology and algorithm of data mining can be used for mining, it is very likely to understand the causes of students' problems at a deep level. For this purpose, it is necessary to discover the accumulated large amount of student psychological assessment data. The process of psychological assessment of college students is shown in Figure 3. Psychological quality is also an essential part of students' quality and has a constraining effect on the cultivation and development of students' quality. The starting point and focus of conducting psychological quality research are to improve the overall quality of students.

### 4.4. Construction and Implementation of a Big Data-Based Psychological Quality Assessment Model for College Students

To ensure the smooth construction of the designed big data analysis-based psychological quality assessment system for college students. This paper will test various functions of the assessment system, build the corresponding psychological quality education platform, objectively and realistically simulate the whole process of online learning and training management. In this paper, we test the application functions of the psychological quality education course management system and gain experience for implementing the project. In this paper, we mainly think from the user's point of view during system testing, so we have to find the product's defects first and adjust them in time during testing the product.

The content of this system test is mainly divided into two parts: function and performance, after comparing with other course management systems to obtain the system test results and reflect the operational advantages of this system.

The operating environment for designing the psychological assessment management system can be divided into server-side and client-side. The server-side uses XEON dual CPUs and ensures more than 2 GB of memory. A database system is embedded in the server-side to store all the data generated during the system's operation. The client-side is an ordinary PC with Internet Explorer 6/Opera/Firefox and other mainstream browsers. The server and the client are installed in a wireless communication network environment with 2 Mb/s bandwidth.

Set the test contents of the system for course management function and system running performance, respectively, set the operation task and expected output result of course management, and compare the actual impact of the system running output with the desired effect to judge the success rate system management function. The system function's running time is called to realize the comparison of the system course management efficiency [26]. And the system operation performance test index for the system's compatibility, different universities psychology students use various quality education equipment. Therefore, the designed system needs to ensure operating in various experimental environments. Calculating the number of runnable equipment in the number of experimentally prepared devices was used to derive quantitative comparison results of system compatibility. Psychological qualities are based on physiological conditions, internalize externally acquired stimuli into stable, essential, and implicit, have primary, derivative, developmental and self-organizing functions, and are closely connected with the adaptive, developmental, and creative behavior of a person. To form an experimental comparison, in addition to the designed data mining-based course management system for psychological education of college students, a traditional course management system and a Java EE-based technology proposed in the literature were set up. Through functional runs and statistics, it was found that both the conventional method and the course management system proposed in the literature had problems such as no CAPTCHA for login, poor user interaction, and course addition failure. The comparative results of assessment management efficiency in terms of running time are shown in Figure 4.

## 5. Discussion

To effectively improve the psychological quality of college students and better play the role of “nurturing” in the mental health education of college students, we need to make efforts and exploration in the following aspects: focus on excavation and give full play to the excellent role of aesthetic education in improving the mental health education of college students. In the ideological and political education work of colleges and universities, the most significant difficulty is how to change the state of passive education of college students and awaken their inner vitality and tension of life. In the operation phase of the extensive data analysis process, the platform-oriented big data analysis process model is instantiated into a process instance that conforms to the execution platform specification according to the analysis module entity corresponding to each node as well as the input and output pattern information and parameter information. As a sure fun and entertainment, aesthetic education can express profound philosophies in an easy-to-understand form and content, which can make college students experience life, feel emotions and understand life in a relaxed and happy state, and have a profound influence on students' life value choice, interpersonal communication, and self-awareness, etc., and cultivate and shape college students' good psychological quality in feeling beauty, cognizing beauty and expressing beauty. It plays a vital role in improving the comprehensive quality of college students.

Good at innovation, give full play to the positive role of new media in mental health education. To better carry out mental health education for college students, colleges and universities, in actively exploring new ways and means of ideological and political teaching, should fully exploit the positive influence of film and television works, variety shows, etc., and through an innovative batch of arts and crafts to meet the needs of engineering education professional certification for students' comprehensive quality improvement; design and use the “student growth handbook.” Adopt the process evaluation and dynamic evaluation to focus on the development and growth of students. Pay attention to the changes in growth and progress and form a classroom teaching evaluation system that incorporates developmental evaluation. The evaluation process can be extended to follow students for life after graduation, creating a closed-loop to continuously revise and improve the model and method of classroom education in colleges and universities.

In this study, the new simplified version of the Psychological Quality Questionnaire for College Students (CSPSz-SV) was analyzed using multiple generalization theories. The study showed a close correlation between the subjects' scores on the three factors of the CSPSz-SV, and there was both relative independence and close correlation among the three factors, which supported the 3-factor structure theory of psychological quality. However, whether the scores of the three factors can be combined into one total score (psychological rate) remains to be determined by the results of the D study. In addition, the variance of the subjects in all three factors was more significant, indicating that the issues and the conflict related to the topics were more critical in the variance of the test scores. Big data analytics is a series of analysis processes aimed at maximizing the value of data for specific domain application scenarios and obtaining valuable decision-making information such as patterns, trends, and correlations implied by them. In contrast, the variance of the test questions was relatively more minor, indicating that the friction caused by the test questions was less critical in the variance of the test scores, which suggested that the quality of the questions in each of the CSPSz-SV factors was good. This indicates that it is feasible to divide the CSPSz-SV into three elements: cognitive quality, personality quality, and adaptability. The measurement properties of the questionnaire are better after extracting the three factors. At the same time, the probability coefficient and reliability index of the global total score of the questionnaire reach the ideal level and are higher than the corresponding index of each factor. The relative error variance and absolute error variance of the global total score are then the related results of each element, so it is feasible and reasonable to combine the scores of the three factors into one total score (psychological quality). It can be better used when combining the three factors into one full scale. The questionnaire can be used on a full scale. Accordingly, when evaluating the psychological quality of college students, it is possible to examine the specific performance of college students in terms of cognition, personality, and adaptability based on the scores of each factor, and it is also possible to use the total score to evaluate the overall psychological quality of college students. Thus, the CSPSz-SV can be used to assess the psychological quality of college students in practice.

Levels can be used for both norm-referenced tests and criterion-referenced tests.

## 6. Conclusion

This paper designs a psychological quality assessment system for college students with the help of big data technology and verifies the effectiveness of the psychological quality assessment system for college students based on extensive data analysis, which makes the management of psychological quality assessment for college students more perfect. In terms of the leading development indicators of college students, there is a significant correlation between college students' psychological quality and psychological health, social adaptation, and academic development. Not only do you need solid theoretical knowledge, but also a healthy body and a good heart. The university stage is critical for most college students to mature physically and mentally gradually. It is also essential for college students to slowly develop from immaturity to maturity. After controlling for the effects of demographic variables, the results of stratified regression analysis show that the psychological quality of college students still has a significant impact on psychological health, social adaptation, and academic development, and the intrinsic functional role of psychological quality varies for different developmental indicators. In general, cognitive quality has significant effects on indicators closely related to academic achievement and personal accomplishment, and insignificant impact on indicators involving emotional-emotional and value judgment; personality quality mostly had a substantial effect on hands involving emotional-emotional state, and weak effects on achievement and accomplishment; adaptability has a significant effect on indicators of mental health, social adaptation, and academic development.

## Figures and Tables

**Figure 1:** Differences in the psychological quality of college students.

**Figure 2:** Big data analysis process processing framework.

**Figure 3:** The process of psychological quality assessment of college students.

**Figure 4:** Comparison results of measuring management efficiency.

**Table 1:** Read and write parameters.

Name	Symbol	Minimum value	Typical value	Maximum value
Count data build time	T_DDR_	1	12	30
Write data build time	T_DSW_	1500	3000	5200
Data hold time	T_H_	160	410	920
Address hold time	T_AH_	30	45	120
Address build time	T_Ab_	35	74	150
Pulse width	T_Pw_	34	65	160
Cycle time	T_C_	54	110	210
Rise/fall time	T_F_ T_R_	30	65	130

## Data Availability

The data used to support the findings of this study are available from the corresponding author upon request.
